The article "Postoperative Nursing and Functional Rehabilitation of Ultrasound Diagnosis of Lower Rotator Cuff Injury" was retracted in 2023. Reasons: unreliable results or conclusions; lack of ethics approval or compliance; concerns about the data; concerns about the peer review.

# Postoperative Nursing and Functional Rehabilitation of Ultrasound Diagnosis of Lower Rotator Cuff Injury

**DOI:** 10.1155/2022/8319082

**Published:** 2022-08-28

**Authors:** Riying Hou

**Affiliations:** College of Gerontic Education, Jilin Open University, Changchun, Jilin 130022, China

## Abstract

In order to explore the postoperative nursing effect and functional rehabilitation of rotator cuff repair under ultrasound diagnosis, a method of nursing and rehabilitation functional training for athletes' wrist injury under the assistance of microscopic B-ultrasound was proposed. This study retrospectively analyzed the therapeutic effect of tendon anastomosis in 237 patients with wrist tendon injury, adopted nursing measures such as health education and functional exercise, and observed its clinical effect. The results showed that after 3-6 months of follow-up, all patients had satisfactory recovery of tendon function. Of these, 132 patients recovered well. 84 patients recovered well. The excellent and good rate of patients was 91%. Ultrasound diagnosis of rotator cuff repair combined with functional exercise promotes good recovery of shoulder joint function in patients.

## 1. Introduction

B-ultrasound is a commonly used medical equipment in hospitals. It utilizes the characteristics of ultrasonic wave, such as excellent directivity, strong penetration ability, and obvious reflection characteristics. According to the basic situation of the recovery of ultrasonic signal, it completes ultrasonic imaging by using the recovery part of acoustic signal. Hospital B-ultrasound can complete the diagnosis and observation of diseases, providing a basis for pathological diagnosis and treatment. And it has the characteristics of simple, painless diagnosis, low diagnosis cost, and high acceptance by patients [1].

Wrist joint is one of the joints with the most complex structure and the most frequent movement in the human body, which is also an organ necessary for people to complete daily work. The wrist joint is mainly composed of the distal ulnar and radial bones, eight carpal bones, and the proximal end of the 1st to 5th metacarpal bones. The complex motion is usually accomplished by the cooperation of the ulnar deflection force, the dorsiflexion force, and the rotation force. The three forces affect each other and easily cause the injury of bone, cartilage, and soft tissue. Therefore, wrist injuries are mostly mixed injuries, often multiple wrist fractures, joint dislocation, and soft tissue edema. Wrist joint injury is a common and frequently occurring clinical disease. If it cannot be treated timely and accurately, it is easy to lead to wrist joint function and activity disorders. Therefore, accurate diagnosis of wrist joint injury is particularly important. Imaging examination plays an important role in wrist joint injury and is the most important auxiliary diagnosis method, which can provide clinicians with clear and intuitive image information and provide reliable basis for subsequent clinical treatment plan. X-ray is the preferred clinical method in the imaging examination of wrist joint injury, but its two-dimensional image has some limitations in the imaging diagnosis, which is prone to misdiagnosis and missed diagnosis. In recent years, multislice spiral CT (MSCT) and nuclear magnetic resonance (MRI) techniques have been widely used to improve the accuracy of wrist injury imaging diagnosis. With the improvement of ultrasound technology and the improvement of sensitivity, the application of ultrasound in wrist joint injury has been further expanded [2].

The article "Postoperative Nursing and Functional Rehabilitation of Ultrasound Diagnosis of Lower Rotator Cuff Injury" was retracted in 2023. Reasons: unreliable results or conclusions; lack of ethics approval or compliance; concerns about the data; concerns about the peer review.

X-ray has the advantages of simple operation and low price, which is widely used in the diagnosis of tumors and bone and joint injuries. It can clearly display fracture and joint dislocation, which has always been the preferred imaging examination method for wrist joint injuries. Patients with wrist trauma are routinely diagnosed by X-ray anteropostery and lateral radiography. Changes in the morphology of some wrist joints on radiographs suggest abnormalities in the wrist joint. For example, there are “three arcs” in the wrist joint, namely, the two arcs on the far and far sides of the scaphoid bone, lunate bone, and deltoid bone and the arc on the proximal articular surface of the head and scaphoid bone on the orthographic film. Changes in any one of the arcs indicate joint abnormalities. The width of the wrist joint space is basically the same, 1 ~ 2 mm. If the joint space narrowed or even disappeared, indicating the possibility of dislocation. The lunate bone is located in the middle of the articular surface of the distal radius on the lateral radiographs and is basically quadrilateral on the anteroposteric radiographs. If the shape and position of the lunate bone change significantly, it suggests the occurrence of lunate bone dislocation. On lateral wrist radiographs, lunate bone, skull, and radial longitudinal axis should be basically in a straight line, and severe deviation would be considered as dislocation [3]. The change of “triangle shadow” has important diagnostic value for most carpal dislocation. The determination of “tear drop angle” on X-ray lateral film is instructive to the determination of step and fissure of articular surface. It is important to remember that the measurement of length and width is helpful to analyze the changes and damage degree of radial sigmoid notch. Parameters such as the width of the distal radius are helpful for diagnosing the degree of articular surface injury and wrist instability. Dorsal deltoid fractures can be diagnosed by clinical manifestations combined with lateral wrist radiographs. “Terry-Thomas sign” and “overflow cup sign” are helpful for the early and late diagnosis of perilunate dislocation, respectively. The anatomical structure of wrist joint is complex, the shape of carpal bone is diverse, and the injury situation is also complex and diverse. In addition to fracture or fracture accompanied by dislocation, there can be structural disorder and deformity. If accompanied by soft tissue swelling, bleeding gauze wrapping, etc., it will form interference to the examination. There are still many deficiencies in the diagnosis of wrist joint injury by X-ray plain film. For complex fractures or multiple fractures, many hidden fractures and microfractures are often missed and misdiagnosed due to overlapping. Although X-ray is the first choice in clinical examination of ulna impingent syndrome, it cannot accurately diagnose the patients with early ulna impingent syndrome. X-ray has low sensitivity in the diagnosis of lunate dislocation and perilunate dislocation, which is easy to be missed and misdiagnosed. The probability of missed diagnosis and misdiagnosis is also high for dorsal fracture of the wrist triangle bone. Patients with wrist trauma are usually in passive position. And it is often difficult to take the standard projection position due to pain, which leads to carpal bone overlap and deformation, affecting the accuracy of diagnosis. In the case of wrist plaster external fixation, accurate diagnosis is more difficult [4].

The article "Postoperative Nursing and Functional Rehabilitation of Ultrasound Diagnosis of Lower Rotator Cuff Injury" was retracted in 2023. Reasons: unreliable results or conclusions; lack of ethics approval or compliance; concerns about the data; concerns about the peer review.

Ultrasonic examination, which is widely used in tumor, cardiovascular, oral, and other diseases, has the advantages of safety, speediness, no radiation, and so on. With the improvement of ultrasonic technology, its sensitivity has been continuously improved, further expanding the application of ultrasonic examination in wrist joint injury and reducing the dependence of wrist joint lesions on CT and MRI. As shown in Figure 1, the Ultrasound Institute and the Radiological Society recommend the use of a broadband, high-resolution ultrasound probe for wrist examination due to the relatively shallow position of the wrist. This probe can obtain better images, which is helpful for doctors to observe wrist joint injury. Ultrasound examination of wrist joint injury can not only be used to evaluate the traumatic injured muscles, tendons, ligaments, and peripheral nerves but also clearly display joint effusion [5]. The use of 3D ultrasound provides more images of normal and abnormal tissues than conventional two-dimensional ultrasound, allowing for more evaluation of damage. Ultrasound can clearly show the adjacent situation of the tissues such as blood vessels and nerves around the wrist and some soft tissue lesions such as tendinitis, tenosynovitis, bursitis, tenosynovitis, ganglion cyst, joint effusion, nerve compression, and injury. The diagnosis of injury tenosynovitis is convenient and fast. High-frequency ultrasound can accurately display and diagnose TFCC injury and bone erosion in patients with early and active rheumatoid arthritis (RA), which can be applied to the diagnosis and follow-up of RA. Combined with angiography, it can also conduct qualitative and semiquantitative analysis of RA synovial blood perfusion [6].

The article "Postoperative Nursing and Functional Rehabilitation of Ultrasound Diagnosis of Lower Rotator Cuff Injury" was retracted in 2023. Reasons: unreliable results or conclusions; lack of ethics approval or compliance; concerns about the data; concerns about the peer review.

However, the penetration of ultrasound is weak, and the anatomical structure of the carpal bone cannot be completely and clearly displayed by ultrasound examination. In addition, the compression of the ultrasonic probe will cause discomfort in patients with wrist trauma, etc., and there are still some limitations in the examination of wrist injury.

To sum up, different imaging examination methods have their own advantages and disadvantages in wrist joint injury. If a single examination is used for analysis and diagnosis, missed diagnosis and misdiagnosis may often occur.

## 2. Literature Review

Sagar et al. proposed the theory of wave-particle duality, believing that the motion of electrons is similar to the propagation of visible light [7]. Taa et al. proposed the motion theory of electron in magnetic field and pointed out that the magnetic field with axial symmetry has the effect of deflection and focusing on electron beam [8]. The discovery of wave-particle duality theory and magnetic focusing theory provides important theoretical guidance for the invention of electron microscope. Using electron beam instead of visible light as illumination source can greatly improve the geometric resolution and effective magnification of electron microscope, which is an important basis for the existence of electron microscope. Ashkenazi et al. confirmed the possibility of electronic imaging for the first time and obtained an electronic image of copper net magnified 12 times [9]. Subsequently, with the joint efforts of El-Rosasy and Ayoub, transmission electron microscopy of commodities was developed and gradually popularized [10]. The resolution of Elmiskop I transmission electron microscope developed by Mc et al. was better than 1 nm [11]. Chi et al. first proposed the principle and design idea of scanning electron microscopy [12]. On the basis of the secondary electron detector designed and improved by Mlha et al., the first practical scanning electron microscope was specially developed for the Canadian Pulp and Paper Research Institute, which made a great contribution to the development of modern scanning electron microscopy and was in the National Science Museum of Canada [13]. Ncha et al. made the first commercial scanning electron microscope of model Mark I [14]. The secondary electron detector (ET-D) improved and perfected by Chen et al. had also become a necessary secondary electron detector for all current scanning electron microscopy [15]. At the end of 1980s, Lotzien et al. successfully developed the environmental scanning electron microscope and began to sell them [16].

The article "Postoperative Nursing and Functional Rehabilitation of Ultrasound Diagnosis of Lower Rotator Cuff Injury" was retracted in 2023. Reasons: unreliable results or conclusions; lack of ethics approval or compliance; concerns about the data; concerns about the peer review.

Improving the image quality and resolution of electron microscope was the direction of continuous efforts of scientists and electron microscope engineers all over the world. In terms of electron emission sources, tungsten filament cathode had gradually developed to lanthanum hexaboride cathode and then to high resolution field emission cathode. Field emission cathodes could be divided into cold field and hot field, respectively. The electron energy divergence of the cold field emission cathode was smaller, and the current density was larger. Although the electron energy divergence of the hot field emission cathode was slightly larger than that of the cold field and the current density was slightly smaller than that of the cold field, the total emission current of the hot field emission cathode was larger, the stability was better, and the anti-interference ability was stronger. In the electronic imaging technology, Americans invented the eight pole astigmatism device and then gradually invented the spherical aberration correction device, monochromator, and other parts which helped to improve the resolution of the image. In terms of image recording media, the traditional photosensitive film mode had been replaced by the CDD camera mode, and more advanced CMOS cameras had been gradually popularized and used [17]. With the continuous development and deepening of these new technologies, the current highest resolution of transmission electron microscopy and scanning electron microscopy had reached the high level of 0.07 nm and 0.4 nm, respectively [18].

In addition, energy dispersive spectrometer, spectrograph, EBSD, FIB, freezing technology, and 3D reconstruction technology have also developed rapidly in recent decades [19]. The combination and integration of these techniques with the electron microscope greatly enhance the detection function and analytical ability of the electron microscope.

## 3. Methods

### 3.1. Surgical Methods

In previous literature, brachial plexus block anesthesia was performed with the patient in supine position. The shoulder joint was placed on the side table with the extension 90°. The index finger, middle finger, and ring finger were put into the traction finger sleeve. Traction tower was used to tract the radial fracture end longitudinally. After the C-arm perspective was satisfying, the fracture end was fixed by a 1.5 mm Kirschner wire at the styloid process of the radius, and the finger sleeve was removed from the traction tower. The forearm was horizontally positioned. The skin and fascia were longitudinally cut between the flexor carpi radialis tendon and radial artery. The anterior rotator muscle was cut from the radial insertion to expose the extra-articular fracture. If the traction reduction was not satisfactory, the Kirschner wire could be withdrawn to the distal side of the fracture, and the finger press could be used to continue the Kirschner wire after the reduction was satisfactory [20]. The plate was placed close to the volar side of the radius. After the adjustment of the lower C-arm was satisfied, the plate was fixed with ordinary compression screws through the sliding hole to make it close to the radius, and then the locking screws on the lower part of the ordinary nail were inserted. Again, the traction finger sleeve was hung on the traction tower for traction, and the traction force was 5-7 kg. It approached on 3/4 and 4/5 of the dorsal side of the wrist joint, each about 0.3 cm long. And the arthroscope and plane were inserted to attract the blood stasis in the joint and make the field of vision clear [21]. The radial articular surface and surrounding ligaments were observed. Kirschner wire and probe hook were used to pry the joint fracture block to make it smooth. The joint space was less than 1.0 mm, and the joint step was less than 1.0 mm. Kirschner wire was used to fix temporarily. After C-arm fluoroscopic reduction was satisfactory, the plate distal screw was placed. Arthroscopy was used to assist to observe whether the screw entered the articular cavity and whether the length of the screw penetrated out of the dorsal bone cortex. The traction device was removed, the wound was rinsed, the radial edge of the anterior muscle was sutured, and the subcutaneous and skin were sutured. Posterior external fixation was assisted for C3 distal radial fractures. And antirotation flexion and extension bracing was assisted for C1 and C2 distal radial fractures complicated with TFCC injury.

The article "Postoperative Nursing and Functional Rehabilitation of Ultrasound Diagnosis of Lower Rotator Cuff Injury" was retracted in 2023. Reasons: unreliable results or conclusions; lack of ethics approval or compliance; concerns about the data; concerns about the peer review.

### 3.2. Nursing Methods

#### 3.2.1. Postoperative Day Care

Postures care were taken immediately after patients entered the ward after surgery. The affected limb was placed on a 30° elevation pad to ensure that the wrist was about 10.0 cm higher than the heart level. At the same time, psychological counseling was carried out to eliminate patients' tension. According to the surgical records, the patients and their families were instructed about the precautions for the affected limb, and the pamphlet *Early Rehabilitation Guide for Arthroscopic Treatment of Distal Radius Fracture* was issued. The injured wrist was wrapped with a medical ice pack to help stop bleeding and detumation and prevent compartment syndrome. Anti-infective and detumescent drugs were administered intravenously [22].

#### 3.2.2. 2 ~ 7 Days Postoperative Nursing

On the 2nd day after surgery, patients could get out of bed and carried out rehabilitation training of shoulder, elbow, and finger, especially the inflexible flexor tendon caused by the stimulation of surgery and steel plate. Early finger flexion and extension training were beneficial to prevent tendon adhesion and joint stiffness. The six-step method was used for training. Because the flexor thumb tendon was located in the deepest layer and the plate was the largest, the thumb could be used for opposite finger and opposite palm training to the other four fingers in the early stage. At the same time, thumb dorsiflexion, adduction, and abduction training could be conducted, with 30 min each time and 6 times a day.

#### 3.2.3. 7 ~ 14 Days Postoperative Nursing

On the 7th day after surgery, early health equipment (grip ball, grip machine, finger extension and flexion trainer, etc.) could be assisted. Passive wrist flexion and extension training could be used for non-C3 distal radius fractures, with passive flexion and extension ranging from -10° to 10° at week 1 and passive flexion and extension ranging from -20° to 20° at week 2. Patients were encouraged to perform active wrist flexion and extension training after passive flexion and extension. Patients without TFCC injury could passively train pronation and supination movements [23].

#### 3.2.4. 3~6 Weeks Postoperative Nursing

Postoperative 3 weeks of wrist range of motion were -30°~30°, and postoperative 4 weeks of wrist range of motion were -40°~40°. At the same time, the strength training was strengthened. At this time, auxiliary grip and pinch force training could be conducted. Patients without TFCC injury could be passively trained in pronation and supination. Five to six weeks after the operation, patients could take active training, with the forearm placed on the flat table and wrist joint located at the table. And when the healthy hand assisted pulling the affected wrist, flexion and extension training were conducted at the same time [24].

The article "Postoperative Nursing and Functional Rehabilitation of Ultrasound Diagnosis of Lower Rotator Cuff Injury" was retracted in 2023. Reasons: unreliable results or conclusions; lack of ethics approval or compliance; concerns about the data; concerns about the peer review.

#### 3.2.5. 7~8 Weeks Postoperative Nursing

At the 7th week after surgery, wrist weight-bearing drafting was started, starting with 0.5 kg weight-bearing and progressing step by step. At this time, the brace was removed for patients with TFCC injury, and passive pronation and supination training were conducted. Passive wrist flexion and extension and lateral deflection training were performed. The activity limit remained 10-20 s. The patient was instructed to carry out fine motor coordination exercises, such as writing, typing on the keyboard, and twisting bottle caps. At the 8th week after surgery, muscle strength training and resistance training of wrist joint and forearm were mainly started. At this time, flexion, extension, pronation, supination, and ulnar deviation were trained with rubber strips with different elastic forces [25].

## 4. Experiment Results and Discussions

In previous literature and general data, 237 patients with hand tendon injury were selected, including 150 males and 87 females. The age ranged from 18 to 83 years, with an average age of (41.6 ± 11.4) years. There were 180 cases of cutting injury, 20 cases of smashing, 17 cases of rolling, 5 cases of fracture complication, and 15 cases of strangulation. Of the 237 patients, 12 had edema, 5 had tendon adhesion, 2 had tendon rupture, and 2 had joint stiffness after surgery, see Figures 2–5, Table 1.

The patients were followed up for 3-6 months. All the 237 patients had satisfactory recovery of tendon function. 132 patients had excellent recovery. 84 patients had good recovery. 11 patients had moderate recovery. And 10 patients had poor recovery. The rate of excellent and good treatment was 91%.

Hand is an important tool in daily life and work, which plays an important role in life and work. With the development of economy, people's living standards have improved significantly, and their expectation for treatment is increasing. For hand trauma patients, functional recovery of the affected finger after operation is not only simple morphological repair but more attention is paid to the effect of functional modification. And the medical concept is also changed from simple surgical treatment to rehabilitation treatment. Postoperative nursing and functional exercise guidance are particularly important after hand tendon injury. Proper treatment can reduce complications such as tendon adhesion and joint stiffness and maximize the maintenance of hand function.

To sum up, hand tendon injury nursing is a comprehensive, systematic, and effective nursing method, which is mainly through improving patients' awareness of disease knowledge to effectively improve the symptoms of patients and promote the rehabilitation of patients ultimately.

The article "Postoperative Nursing and Functional Rehabilitation of Ultrasound Diagnosis of Lower Rotator Cuff Injury" was retracted in 2023. Reasons: unreliable results or conclusions; lack of ethics approval or compliance; concerns about the data; concerns about the peer review.

## 5. Conclusion

In the research, a method of nursing and rehabilitation function training of athletes' wrist joint injury assisted by microscope B-ultrasound was proposed. The method was as follows. Brachial plexus block anesthesia was performed with the patient in supine position. The shoulder joint was placed on the side table with the extension 90°. The index finger, middle finger, and ring finger were put into the traction finger sleeve. Traction tower was used to tract the radial fracture end longitudinally. After the C-arm perspective was satisfying, the fracture end was fixed by a 1.5 mm Kirschner wire at the styloid process of the radius, and the finger sleeve was removed from the traction tower. The nursing method of nursing and rehabilitation measures was taken from the beginning to the seventh or eighth week after surgery. The patients were followed up for 3-6 months by retrospective analysis and observation. All the 237 patients had satisfactory recovery of tendon function. 132 patients had excellent recovery. 84 patients had good recovery. 11 patients had moderate recovery. And 10 patients had poor recovery. The rate of excellent and good treatment was 91%. It proved the effectiveness of the experience of nursing and rehabilitation function of athletes' wrist joint injury assisted by microscope B-ultrasound. In the future, it is believed that more and more cases of nursing and rehabilitation function exercise of athletes' wrist injury will be completed with the help of microscope and B-ultrasound.

## Figures and Tables

**Figure 1:** Athlete's wrist injury assisted by B-ultrasound.

**Figure 2:** Comparison of minimum indexes of lung function in the control group.

**Figure 3:** Comparison of maximum indexes of lung function in the control group.

**Figure 4:** Comparison of minimum indexes of lung function in the treatment group.

**Figure 5:** Comparison of maximum indexes of lung function in the treatment group.

**Table 1:** Comparison of average hospitalization expenses and days in the hospital between the two groups (*x* ± *s*).

Group	Cases	Hospitalization expenses	Days in hospital
The treatment group	119	4068.91 ± 746.32	11.12 ± 2.14
The control group	118	5176.39±	14.93 ± 3.21
*t*		4.92	3.09
*P*		0.001	0.003

## Data Availability

The data used to support the findings of this study are available from the corresponding author upon request.
